# COPS3 Promotes Proliferation, Invasion, and EMT of Colorectal Cancer Cells by MEK/ERK Pathway

**DOI:** 10.1155/2022/7594489

**Published:** 2022-07-19

**Authors:** Yanchao Xie, Zhijiang Wei, Chi Cheng

**Affiliations:** Department of Gastroenterology, Cangzhou Central Hospital, Cangzhou, Hebei 061000, China

## Abstract

Colorectal cancer (CRC) is one of the most aggressive cancers with poor prognosis and high mortality. The study of the pathogenesis of CRC is a top priority in providing effective diagnostic and prognostic strategies for CRC. COPS3 protein is a subunit of the COP9 signaling body (CSN), which is closely associated with the development of multiple types of tumors. However, there are few studies on the role of COPS3 in colon adenocarcinoma (COAD). This study investigated the effects of COPS3 on proliferation, motility, and EMT of colorectal cancer cells and related mechanisms. COPS3 was highly expressed in COAD. The depletion of COPS3 suppressed the viability and stimulated the apoptosis of COAD cells. Depletion of COPS3 suppressed the motility and EMT process of COAD cells. Mechanically, we found that COPS3 could mediate MEK/ERK pathway and therefore affected the process of COAD cells. We thought that COPS3 could serve as a promising COAD target.

## 1. Introduction

Colorectal cancer (CRC), as one of the most aggressive cancers with poor prognosis, causes a large number of deaths worldwide and affects millions of people every year [1, 2]. CRC mainly affects the distal rectum, sigmoid colon, and descending colon [3]. More and more CRC risk factors have been reported recently, such as ageing, unhealthy diet, smoking, obesity, physical inactivity, inflammatory bowel disease, and genetic factors [4]. Treatment for CRC includes surgery, chemotherapy, and radiotherapy [5, 6]. However, because the detailed mechanism of CRC development is not fully understood, the 5-year survival rate for CRC is low, especially in the later stages [7]. Therefore, a better understanding of the pathogenesis of CRC is a top priority in providing effective diagnostic and prognostic strategies for patients with CRC.

COPS3 protein is a subunit of the COP9 signaling body [8], located in chromosome region 17p11.2 and plays a role in deubiquitination and protein kinase activity in a variety of processes [9]. COPS3 is closely associated with tumor development [10, 11]. Knockdown of COPS3 significantly reduced lung metastasis of osteosarcoma cells in mouse models, downregulated MEK and ERK signaling, and inhibited EMT by 90 kDa ribosomal S6 kinase (RSK), reducing metastasis of osteosarcoma cells [12]. In addition, COPS3 depletion inhibited tumor growth in nude mice by blocking cell cycle progression [13]. However, there are few studies on the role of COPS3 in colorectal cancer, particularly colon adenocarcinoma (COAD).

MEK/ERK cell signaling pathway plays an important role in various human tumors and is involved in cell proliferation, survival, metabolism, and cell migration [14]. For example, sophorine inhibits tumorigenesis in colorectal cancer by downregulating the MEK/ERK/VEGF pathway [15]. Epithelial mesenchymal transformation (EMT) is a biological process in which cancer cells lose their epithelial features and acquire mesenchymal markers, which make tumor cells more mobile and invasive [16]. EMT is marked by decreased E-cadherin expression and increased N-cadherin or Vimentin expression [17]. The process of EMT is controlled by transcription factors and certain pathways.

This study investigated the effects of COPS3 on proliferation, migration, invasion, and EMT of colorectal cancer cells and related mechanisms. Our data revealed that COPS3 was highly expressed in human COAD cells and affected the viability, motility, and EMT of COAD cells via MEK/ERK pathway. We thought that COPS3 could serve as a promising COAD target.

## 2. Materials and Methods

### 2.1. Antibodies, Primers, and Plasmids

The antibodies used were anti-COPS3 (1 : 500 dilution, ab231344, Abcam), anti-E-cadherin (1 : 1000 dilution, ab76055, Abcam), anti-N-cadherin (1 : 1000 dilution, ab76011, Abcam), anti-Vimentin (1 : 500 dilution, ab8978, Abcam), anti-MEK (1 : 1000 dilution, 178876, Abcam), anti-p-MEK (1 : 1000 dilution, ab278564, Abcam), anti-ERK (1 : 1000 dilution, ab184699, Abcam), anti-p-ERK (1 : 500 dilution, ab201015, Abcam), and anti-*β*-actin (1 : 2000 dilution, 60008-1-Ig, Proteintech).

The quantitative PCR primer sequences of COPS3 are forward, 5′-GCGAGGAAUUGGCAUCCUUTT-3′ and reverse, 5′-AAGGAUGCCAAUUCCUCGCTT-3′. The quantitative PCR primer sequences of GAPDH are 5′-TCCGCCGTGTGTACGTCATT-3′ and 5′-TCCGCCGTGTGTACGTCATT-3′.

siRNA of COPS3 and control siRNA was bought from Riobio (China).

### 2.2. Cell Culture

The normal cell line NCM460 and 4 COAD cell lines, including SW480, HCT116, LoVo, and DLD-1, were all purchased from ATCC. Both of the cells were maintained in DMEM, supplemented with 10% of fetal bovine serum, and incubated at 37°C in a 5% CO_2_ incubator.

### 2.3. Immunoblot Assay

The samples were lysed with the lysis buffer (RIPA, Beyotime, China) and then separated by a 10% SDS-PAGE experiment; sequentially, the total proteins were transferred onto PVDF membranes (Millipore, USA). Then, the PVDF membranes were blocked by the use of 5% dry milk in TBST buffer and antibodies. After washing with TBST for 3 times, the membranes were treated with the secondary antibodies for 45 min. Each blot was then visualized using the ECL kit (GE, SA).

### 2.4. Cell Viability Assays

For CCK-8, COAD cells were plated into the 96-well plates (1000 cell per well) and maintained in complete growth media for 24 h at 37°C. The cells were exposed to CCK-8 reagent at 37°C for 1.5 h. The relative cell viability was assessed with microplate spectrophotometer at 450 nm (Bio-Rad, U.S.A.).

For colony formation assay, COAD cells were plated into 24-well plates (1000 cell per well) and maintained in complete growth media for 14 d at 37°C. Subsequently, the cells were incubated with 0.2% crystal violet and washed, and then, the cells were photographed by a fluorescence microscope (Zeiss, Germany).

### 2.5. Cell Apoptosis Assay

The cells after transfection for 48 h were washed with PBS. Subsequently, the cells were fixed with precooled 70% ethanol at -20°C for 1 h. Subsequently, the cells were stained with propidium iodide (PI) and FITC-labelled Annexin V at 4°C for 10 min, and the apoptosis levels were measured by BD FACS caliber.

### 2.6. Tumor Growth In Vivo Assay

All experimental procedures were according to the criteria outlined in the Regulations of Experimental Animal Administration (http://www.most.gov.cn). Female BALB/c nude mice (8-week-old; weight, ~20 g) were obtained from Beijing Vital River Laboratory Animal Technology Co., Ltd. None of the mice died during the study. A total of 10 athymic nude mice were randomly divided into control (*n* = 5) and transfection (*n* = 5) groups. HCT116 cells which were stably transfected with shRNA plasmids were injected into the right flank of female nude mice. After 2 weeks, the volume of tumors was estimated every week, and the tumor growth curves of 7 consecutive weeks were calculated. The final tumor volume was calculated according to the equation: Tumor volume (mm^3^) = tumor length (mm) × tumor width (mm)2/2.

### 2.7. Statistics

Data were represented as mean ± SD. The statistical significance of the difference was evaluated by Student's *t* test, and *p* < 0.05 was considered significant.

## 3. Results

### 3.1. COPS3 Was Highly Expressed in COAD

We first detected the expression levels of COPS3 in COAD tissues through the analysis in TCGA database. We noticed that the transcript per million of COPS3 in primary tumor tissues (*n* = 286) was higher than normal (*n* = 41), suggesting the high expression in COAD (Figure 1(a)). COPS3 mRNA level increased, indicating that COPS3 high expression may be transcriptional. We then detected the expression of COPS3 in normal cell line NCM460 and 4 COAD cell lines, including SW480, HCT116, LoVo, and DLD-1, through qPCR and immunoblot assays. We found that COPS3 was highly expressed in COAD cell lines at mRNA and protein levels (Figures 1(b) and 1(d)). We therefore thought that COPS3 was highly expressed in COAD.

### 3.2. COPS3 Depletion Suppressed the Viability of COAD Cells and Stimulated Apoptosis

Then, the effects of COPS3 on the viability and apoptosis of COAD cells were evaluated by the transfection of its siRNA in COAD cells including SW480 and HCT116. qPCR and immunoblot confirmed that the transfection of its siRNA decreased the expression of COPS3, compared to the control and NC-siRNA groups in these cells at mRNA and protein levels (Figures 2(a) and 2(b)). Through CCK-8 assays, we found that COPS3 ablation decreased the OD value at 450 nm wavelength, suggesting the inhibition of cell viability (Figure 2(c)). Further through colony formation, we found that the knockdown of COPS3 also decreased colony number in SW480 and HCT116 cells (Figures 2(d) and 2(e)). In addition, FCM assays showed that the depletion of COPS3 contributed to the apoptosis of SW480 and HCT116 cells, with the increased percentage of apoptosis cells (Figures 2(f) and 2(g)). We further detected the expression of cleaved caspase-3 and Bcl-2 in control and COPS3 siRNA cells and further confirmed the previous conclusion (Figure 2(h)). Therefore, COPS3 depletion suppressed the viability of COAD cells and stimulated apoptosis.

### 3.3. The Knockdown of COPS3 Suppressed the Motility of COAD Cells

We then detected the effects of COPS3 on the motility of COAD cells. We found that its ablation increased the wound width at 24th hour time point, in SW480 and HCT116 cells (Figures 3(a) and 3(b)). We therefore thought depletion of COPS3 suppressed COAD cell migration. Further, we found its knockdown suppressed the invasion of SW480 and HCT116 cells, with the decreased number of invasive cells (Figures 3(c) and 3(d)). Therefore, COAD3 knockdown inhibited the motility of COAD cells.

### 3.4. Knockdown of COPS3 Suppressed the EMT in COAD Cells

Since previously we showed the effects of COPS3 on COAD3 cell viability and migration, we then investigated its role in the COAD cell EMT process. We detected the expression of several EMT markers. Through immunoblot assays, we found that COPS3 knockdown increased the protein levels of E-cadherin and downregulation of N-cadherin and Vimentin, in both SW480 and HCT116 cells (Figure 4). Therefore, depletion of COPS3 suppressed the EMT process in COAD cells.

### 3.5. COPS3 Mediated the MEK/ERK Pathway in COAD Cells

Then, we investigated the possible mechanism underlying COPS3 affecting COAD progression. The previous study indicated the effects of COPS3 on the MEK/ERK pathway, which could mediate the proliferation, motility, and EMT in several types of tumor cells [12]. We then detected whether COPS3 could mediate this pathway in COAD cells. Through immunoblot assays, the knockdown of COPS3 decreased the phosphorylation levels of MEK and ERK in both SW480 and HCT116 cells (Figure 5). Therefore, we thought COPS3 could mediate the MEK/ERK in COAD cells.

### 3.6. COPS3 Depletion Suppressed Tumor Growth *In Vivo*

To further confirm whether COPS3 deficiency was able to repress tumor growth, the in vivo assays were constructed. Through injection of COPS3 deficiency HCT116 cells into nude mice, we measured and calculated the growth curves of tumors. Consistent with our hypothesis, the volumes of tumors in COPS3-depleted groups were markedly smaller than the negative control groups (Figure 6(a)). To ulteriorly identify the silencing efficiency of COPS3 siRNA, we detected the expression of COPS3 in tumor tissues of mice via IHC and immunoblot assays, and the data revealed that compared with the negative groups, the protein levels of COPS3 were efficiently restrained by COPS3 siRNA in the COPS3 depletion groups (Figures 6(b) and 6(c)). We further detected the expression of E-cadherin, Erk, p-Erk, Mek, and p-Mek through immunoblot, and the data further confirmed our previous conclusion (Figure 6(d)). Therefore, COPS3 depletion suppressed tumor growth in vivo.

## 4. Discussion

CRC is a common gastrointestinal malignancy occurring in the colon [18]. CRC inchoate symptom is more not apparent and often already was in progress period when seeing a doctor, right now commonly used remedial measure [2]. To improve the resection rate, reduce the recurrence rate, and improve the survival rate, the treatment of intermediate and advanced CRC is based on surgery, supplemented by chemotherapy, immunotherapy, traditional Chinese medicine, and other supportive therapies [18]. Recently, targeted therapy has made a series of positive progress and has great potential to improve the survival rate of patients with advanced colorectal cancer [19]. However, there are new and more therapeutic targets for the CRC treatment. Here, we noticed that COPS3 was highly expressed in COAD. It affected the viability, motility, and EMT of COAD cells. We thought it could act as a target of COAD.

Through a series of in vitro assays, we concluded that COPS3 was highly expressed in human COAD cells. We further confirmed its effects on the viability, motility, and the process of EMT in COAD cells. COPS3 is an important oncogene involved in metastasis of osteosarcoma [9]. COPS3 depletion could inhibit the growth of lung cancer and liver cancer cells and induce apoptosis [13, 20]. A previous study also revealed that COPS3 played a vital role in linking Raf-1/MEK/ERK pathway and autophagic regulation in osteosarcoma [12]. Depletion of COPS3 could suppress the progression of prostate cancer through reducing phosphorylated p38 MAPK and impairs the EMT [21]. In addition, the overexpression of COPS3 could contribute to the progression of clear cell renal cell carcinoma (ccRCC) via regulation of phospho-AKT, Cyclin D1, and Caspase-3 [22]. The ablation of COPS3 suppressed the proliferation of lung cancer cells via induction of cell cycle arrest and stimulation of apoptosis [13]. These studies with our findings confirmed that COPS3 could serve as a promising target of cancers.

The multiple biological functions of COPS3 have been widely revealed [10]. COP9S3 played a role in regulating mouse oocytes meiosis by regulating MPF activity and securing degradation [23]. The COPS3 is necessary for early embryo survival by way of a stable protein deposit in mouse oocytes [24]. COPS3 is also poised to facilitate communication between the extracellular matrix and the nucleus [25]. Therefore, we guess that COPS3 could induce the deubiquitination of the downstream proteins or the protein kinase activity and therefore mediate the progression of COAD. However, the precise mechanism needs further study.

MEK/ERK signaling pathway can promote the progression of multiple types of cancers, including COAD [26]. The MEK/ERK pathway has been revealed to affect the proliferation, apoptosis, and motility of tumors and affect the EMT progression [12]. Multiple proteins or drugs affected COAD progression via this pathway. For example, Verticillin A could increase the BIM/MCL-1 ratio to overcome ABT-737 resistance in COAD cells by this pathway [27]. These studies all confirmed that MEK/ERK pathway could serve as a promising target of COAD.

In summary, we noticed the high expression of COPS3 in COAD cells. COPS3 contributed to the viability, motility, and EMT of COAD cells via MEK/ERK pathway. We therefore thought COPS3 could serve as a target of COAD.

## Figures and Tables

**Figure 1:** COPS3 was highly expressed in COAD tissues and cell lines. (a) TCGA database showed the levels of transcript per million (TPM) in 286 tumor tissues compared to the 41 normal tissues. (b) qPCR assays showed the mRNA levels of COPS3 in normal cell line NCM460 and 4 COAD cell lines, including SW480, HCT116, LoVo, and DLD-1. (c and d) Immunoblot assays showed the protein levels of COPS3 in normal cell line NCM460 and 4 COAD cell lines, including SW480, HCT116, LoVo, and DLD-1. Data are presented as mean ± SD. ^∗∗^*p* < 0.01 and ^∗∗∗^*p* < 0.001.

**Figure 2:** COPS3 ablation suppressed the viability of COAD cells and stimulated apoptosis. (a) qPCR assays showed the mRNA levels of COPS3 in SW480 and HCT116 cells upon the transfection of control or COPS3 siRNAs or without transfection (control). (b) Immunoblot showed the expression of COPS3 in SW480 and HCT116 cells upon the transfection of control or COPS3 siRNAs or without transfection (control). (c) CCK-8 assays showed the OD value at 450 nm wavelength of SW480 and HCT116 cells upon the transfection of control or COPS3 siRNAs or without transfection (control). (d and e). Colony formation assays showed the colony number of SW480 and HCT116 cells upon the transfection of control or COPS3 siRNAs or without transfection (control). The quantification was in panel (e). (f and g). Flow cytometry (FCM) assays showed the apoptosis percentage of SW480 and HCT116 cells upon the transfection of control or COPS3 siRNAs or without transfection (control). The quantification was in panel (g). (h) Immunoblot showed the expression of the indicated proteins in control or COPS3 siRNAs or without transfection (control). Data are presented as mean ± SD. ^∗∗∗^*p* < 0.001, siCOPS3 vs. siControl.

**Figure 3:** COPS3 knockdown inhibited the migration as well as invasion of COAD cells. (a and b) Wound closure assays showed the wound healing degree of SW480 and HCT116 cells upon the transfection of control or COPS3 siRNAs or without transfection (control). The representative images were shown in (a). The wound width was shown in (b). (c and d). Transwell assays showed the invasive SW480 and HCT116 cells upon the transfection of control or COPS3 siRNAs or without transfection (control). The representative images were shown in (c). The invasive cell number was shown in (d). Data are presented as mean ± SD. ^∗∗^*p* < 0.01 and ^∗∗∗^*p* < 0.001, siCOPS3 vs. siControl.

**Figure 4:** Depletion of COPS3 suppressed the EMT process in COAD cells. Immunoblot assays showed the expression of E-cadherin, N-cadherin, and Vimentin in SW480 and HCT116 cells upon the transfection of control or COPS3 siRNAs or without transfection (control). Data are presented as mean ± SD. ^∗∗^*p* < 0.01 and ^∗∗∗^*p* < 0.001, siCOPS3 vs. siControl.

**Figure 5:** COPS3 mediated the MEK/ERK pathway in COAD cells. Immunoblot assays showed the expression of phosphorylated MEK and ERK and expression of these proteins in SW480 and HCT116 cells upon the transfection of control or COPS3 siRNAs or without transfection (control). Data are presented as mean ± SD. ^∗∗^*p* < 0.01 and ^∗∗∗^*p* < 0.001, siCOPS3 vs. siControl.

**Figure 6:** COPS3 depletion suppressed tumor growth *in vivo*. (a) The representative images of tumors in control and COPS2 siRNA transfection mice and the tumor growth curve. (b) IHC assays showed the expression of COPS2 in tumors in control and COPS2 siRNA transfection mice. (c) Immunoblot showed the expression of COPS2, E-cadherin, Erk, p-Erk, Mek, and p-Mek in tumors from control and COPS2 siRNA transfection mice. Data are presented as mean ± SD. ^∗∗∗^*p* < 0.001, siCOPS3 vs. siControl.

## Data Availability

All data generated or analyzed during this study are included in this published article.
